This article has been retracted.

# TNF-α-induced NF-κB activation upregulates microRNA-150-3p and inhibits osteogenesis of mesenchymal stem cells by targeting β-catenin

**DOI:** 10.1098/rsob.150258

**Published:** 2016-03-02

**Authors:** Nan Wang, Zubin Zhou, Tianyi Wu, Wei Liu, Peipei Yin, Chenhao Pan, Xiaowei Yu

**Affiliations:** 1 Department of Orthopaedic Surgery, Shanghai Jiao Tong University affiliated Sixth People's Hospital, Shanghai, People's Republic of China; 2 Department of Emergency, the first affiliated hospital of Zhengzhou University, Zhengzhou, Henan, People's Republic of China; 3 Department of Orthopaedics and Traumatology, Lui Che Woo Institute of Innovative Medicine, Faculty of Medicine, The Chinese University of Hong Kong, Prince of Wales Hospital, Shatin, Hong Kong SAR, People's Republic of China

**Keywords:** mesenchymal stem cells, β-catenin, TNF-α, microRNA, osteogenesis

## Abstract

Although systemic or local inflammation, commonly featured by cytokine activation, is implicated in patients with bone loss, the underlying mechanisms are still elusive. As microRNAs (miR), a class of small non-coding RNAs involved in essential physiological processes, have been found in bone cells, we aimed to investigate the role of miR for modulating osteogenesis in inflammatory milieu using human bone marrow mesenchymal stem cells (hBM-MSCs). Induced by proinflammatory cytokine TNF-α, miR-150-3p was identified as a key player in suppressing osteogenic differentiation through downregulating β-catenin, a transcriptional co-activator promoting bone formation. TNF-α treatment increased the levels of miR-150-3p, which directly targeted the 3′-UTR of β-catenin mRNA and in turn repressed its expression. In addition, we observed that miR-150-3p expression was increased by TNF-α via IKK-dependent NF-κB signalling. There are three putative NF-κB binding sites in the promoter region of miR-150, and we identified −686 region as the major NF-κB binding site for stimulation of miR-150 expression by TNF-α. Finally, the osteogenic differentiation of hBM-MSCs was inhibited by either miR-150-3p overexpression or TNF-α treatment, which was prevented by anti-miR-150-3p oligonucleotides. Taken together, our data suggested that miR-150-3p integrated inflammation signalling and osteogenic differentiation and may contribute to the inhibition effects of inflammation on bone formation, thus expanding the pathophysiological functions of microRNAs in bone diseases.

## 1. Introduction

A delicate balance between bone resorption and bone formation is required for maintaining the integrity of human bones and physiological functions of the skeletal system, both of which are often disrupted in inflammatory diseases [1–3]. Extensive data have supported that the osteoclast-dependent processes, normally exceeding bone formation during inflammation, are feasible therapeutic targets in treating inflammatory bone diseases with brittle bones [2–4]. In addition, it has received increasing attentions that bone formation activity is also significantly inhibited by inflammatory stimuli. Although the underlying mechanisms are still unclear, the derepression of osteogenesis during inflammation could be potentially used as a valuable strategy to treat patients with osteoporosis, arthritis, Paget's disease or other inflammation-associated bone loss [4,5].

TNF-α is a major proinflammatory cytokine that mediates essential functions associated in bone mass regulation [6]. On the one hand, bone resorption activated by TNF-α has been well characterized [7,8], mediated by the processes such as the increased numbers of osteoclast precursor, enhanced osteoclast differentiation and stimulated osteoclast functional maturation. On the other hand, TNF-α negatively regulates bone formation. It has been suggested that TNF-α can block osteoblast differentiation *in vitro* [9]. In particular, Wnt signalling, a critical pathway driving bone formation, can be repressed by TNF-α [10,11]. The canonical Wnt signalling pathway depends on the stabilization of a transcription cofactor β-catenin [12]. Upon binding to its receptor complex, Wnt protein mainly prevents glycogen synthase kinase 3β (GSK-3β)-targeted β-catenin degradation through the proteasomal machinery. As a result, the accumulation of β-catenin that associates with the Tcf/Lef family of transcription factors in the nucleus directs the expression of canonical Wnt target genes in promoting bone formation [12–14]. The inhibition of Wnt/β-catenin signalling therefore may be directly relevant to the suppressive effects of TNF-α or other proinflammatory cytokines on osteogenic differentiation. Cross-regulations between Wnt and TNF-α signalling have been suggested, and the major downstream player NF-κB activated by TNF-α may mediate the inhibition of Wnt pathway [10,11,15,16]. However, the list of molecular players involved in this process is incomplete.

An important class of candidate gene modulators that have not been explored in this context includes microRNAs (miR). These short lengths of nucleotides expressed from non-coding genome regions specifically target on the 3′ untranslated regions (UTR) of existing mRNAs to attenuate their stability and/or translation efficiency [17]. As an expansion of post-transcriptional control of target genes, microRNAs play multiple functions in regulating bone cell differentiation [18–21]. For example, in C2C12 cells under osteogenic differentiation, multiple miRNAs such as miR-133 and miR-135 that attenuate Runx2 or Smad signalling are downregulated by BMP2 [18]. Conversely, osteoblast lineage differentiation from mesenchymal stem cells also requires the induction of miRNAs such as miR-29, which targets extracellular matrix proteins [20], and the negative regulators of osteogenic differentiation including Wnt signalling [20,21]. The physiological implications of miRNAs like miR-2861 in modulating bone mass in mice and human diseases have also emerged [19]. However, the roles of miRNAs in suppressive effects of inflammation on osteoblast differentiation are unknown, and the identification of specific microRNAs that target Wnt/β-catenin signalling pathway could help to construct a method for the fine-tuning of bone regeneration in therapeutic applications such as inducing bone repair by mesenchymal stem cells.

Here we examined the involvement of microRNAs in osteogenic differentiation during inflammation. Our data pinpointed miR-150-3p as a novel mediator in directing osteogenesis inhibition by TNF-α. We found that miR-150-3p directly targeted the 3′-UTR of β-catenin and blocked its expression. Through a newly identified NF-κB-binding site on the promoter region of miR-150, TNF-α directly stimulated miR-150-3p-dependent reduction of β-catenin in human bone marrow mesenchymal stem cells (hBM-MSCs). These studies established miR-150-3p as a previously unrecognized modulator of osteogenesis in the context of inflammation-associated bone loss, which could be used as a potential therapeutic target for the treatment of related bone abnormalities.

## 2. Material and methods

### 2.1. Human BM-MSC isolation and culture

Ficoll centrifugation (1800*g* for 30 min at room temperature) was used to isolate human bone marrow cells, which were collected from osteotomy sites from patients, who signed informed consent forms. Buffy coat was then carefully collected from the Ficoll-HBSS interface, and washed by HBSS. Viable cells determined by trypan blue exclusion were counted with a haemocytometer and plated at a cell density of 50–100 cells cm^−2^ in 175 cm² flasks or 150 mm dishes. After 24 h, the floating cells were removed, and the adherent cells were cultured at 37°C with 5% humidified CO_2_. Vehicle controls or TNF-α (20 ng ml^−1^) were used to treat the adherent cells for 24 h.

### 2.2. Characterization of hBM-MSC by flow cytometry

Adherent hBM-MSCs were harvested by trypsinization, and the same amounts of cells were resuspended in PBS containing 4% fetal bovine serum. After washing, cells were stained by antibodies that recognize various surface proteins, including CD29, CD90, CD105 and negative marker CD45 (eBioscience). Isotype control antibody-stained cells were used to optimize photo-multiplier tube (PMT) and compensation in the analysis using BD-FACScan. Flow cytometry data were analysed with Flowjo.

### 2.3. MicroRNA-150-3p transfection and measurement

Human miR-150-3p *mir*Vana miRNA mimic and antisense oligos (MH12324) were purchased from Applied Biosystems (Carlsbad, CA, USA), and transfected into cells according to the manufacturer's instructions. Total miRNA was isolated using *mir*Vana miRNA Isolation Kit (AM1561), and expression levels of miR-150-3p were measured with mature miRNA assay kit (478721_mir) and pri-miRNA assay kit (Hs03303271_pri) from Applied Biosystems according to the manufacturer's instructions.

### 2.4. mRNA extraction and real-time PCR

Total RNA was isolated from cell cultures using the RNeasy kit (Qiagen) and was reverse transcribed to complementary cDNAs using Superscript II according to the manufacturer's instructions (Biorad). Specific primers used are shown in table 1. Duplicated PCR reactions were carried out using *n* = 3 for each sample. SYBR Green dye-based detection method was used by using the SYBR Green PCR Master Mix assay (Applied Biosystems). A series of duplicate dilutions of cDNA from control samples were used to optimize the standard curve and validate the melting curves for each primer set.

**Table 1.** Primers used in the study.

PPAR-α	forward primer ATGGTGGACACGGAAAGCC reverse primer CGATGGATTGCGAAATCTCTTGG
ICAM2	forward primer CGGATGAGAAGGTATTCGAGGT reverse primer CACCCACTTCAGGCTGGTTAC
GHR	forward primer CCATTGCCCTCAACTGGACTT reverse primer AATATCTGCATTGCGTGGTGC
CRH-R2	forward primer ATCGGCAAGCTCTACTATGAGA reverse primer TCAGGAGCACGAGAATGATGG
eNOS	forward primer TGATGGCGAAGCGAGTGAAG reverse primer ACTCATCCATACACAGGACCC
β-catenin	forward primer AGCTTCCAGACACGCTATCAT reverse primer CGGTACAACGAGCTGTTTCTAC
Runx2	forward primer TGGTTACTGTCATGGCGGGTA reverse primer TCTCAGATCGTTGAACCTTGCTA
Osterix	forward primer CCTCTGCGGGACTCAACAAC reverse primer AGCCCATTAGTGCTTGTAAAGG

### 2.5. Luciferase assay

Cells were transfected with pGL3 luciferase reporter constructs harbouring the miR-150-3p target sequence of the 3′ UTR of β-catenin (wild-type or mutant sequences). After 24 h, the activities of firefly luciferase and renilla luciferase in the cell lysates were measured with the Dual-Luciferase Assay System (Promega, Madison, WI, USA). For the luciferase transcription reporter assay, miR-150 gene upstream sequences (as indicated) were cloned into the promoter region of the pGL3-Basic vector, and luciferase activity was measured as described above.

### 2.6. Immunoblotting

For the protein analysis of β-catenin protein levels and NF-κB signalling, cultured hBM-MSCs were lysed (10 mM HEPES, pH 7.9, 1.5 mM MgCl_2_, 10 mM KCl, 0.5 mM DTT and 0.2 mM PMSF). Proteins were measured and the same amounts of proteins were then subjected to SDS-PAGE, followed by electric transfer into polyvinylidene fluoride (PVDF) membrane. The antibodies used in Western blot included anti-β-catenin, phosphor-p65 (Ser536) and anti-actin (all from Cell Signaling).

### 2.7. Chromatin immunoprecipitation

Briefly, cultured hBM-MSCs were cross-linked with 1% formaldehyde, sheared to an average size of 400 bp, and subsequently immunoprecipitated with antibodies against NF-κB p65 (Santa Cruz, sc-109). The ChIP-PCR primers were designed to amplify the promoter regions containing putative NF-κB binding sites in the promoter region of miR-150 as illustrated. A positive control antibody (RNA polymerase II) and a negative control non-immune IgG were used to demonstrate the efficacy of the kit reagents (Epigentek Group Inc, P-2025-48). Immunoprecipitated DNA is then cleaned, released and eluted. Eluted DNA can be used for downstream applications of ChIP-PCR. Binding efficiency (Bound/RPII%) was calculated by using a ratio of amplification efficiency of the ChIP sample over polymerase RNA II as 2^(RPII CT – Sample CT)^ × 100%.

### 2.8. Induction of osteoblast differentiation

Osteogenic differentiation of hBM-MSCs was induced by dexamethasone (Dex) (Sigma, USA) in the presence of β-glycerol phosphate and ascorbic acid 2-phosphate [22]. hBM-MSCs after three passages were cultured into a 96-well plate at approximately 80% confluency. The medium was replaced the next day with osteogenic medium (DMEM, 10% FBS, 10 mM glyceraldehydes 3 phosphate, 60 mM ascorbic acid and 10 nM Dex). The osteogenic medium was changed every 2 days.

### 2.9. Alkaline phosphatase staining assay

The hBM-MSCs were cultured and osteogenesis was induced in osteogenic medium. The osteogenic medium was changed every 2 days. At day 8, the cells were analysed. Quantitative analysis was determined by colorimetric assay of enzyme activity. Cells were washed with TB buffer (20 mM Tris, pH 7.5, 150 mM NaCl) twice before being lysed with 100 µl lysis buffer (TB buffer, plus 0.1% Triton). After centrifugation at 12 000 r.p.m. for 20 min at 4°C, 45 µl of supernatant were incubated with 100 µl of ALP substrate *p*-nitrophenyl phosphatate (pNPP) liquid substrate system (Promega, Madison, WI, USA) at 37°C for 20 min, and the absorbance at 405 nm was measured on a 96-well plate reader. The ALP activity was then normalized to the total protein. Imaging analysis was performed in fixed cells stained by freshly prepared 0.1% naphthol AS-MX phosphate, 56 mM 2-amino-2-methyl-1-3- propanediol and 0.1% fast red violet LB salt.

### 2.10. Calcium content assay

Calcium content of the supernatants in cultured hBM-MSCs was measured at day 24 using a Calcium Assay kit (Genzyme Diagnostics, Charlottetown, Canada) following the manufacturer's instructions. Briefly, acetic acid (1 M) was added into the samples and the supernatants were incubated overnight at 4°C for the extraction of the calcium from the mineralized matrix. In a 96-well plate, 15 µl of cell extract was mixed with 150 µl of calcium assay reagent and incubated for 30 s at room temperature. Then the absorbance at 650 nm was measured with a 96-well plate reader. The samples were measured in triplicate and compared with the calcium calibration curve. The calcium content was normalized by cell numbers.

### 2.11. Alizarin red-sulfate staining

For analysing mineralization nodule formation, ALR staining was performed in cells in the osteogenic induction culture for 21 days. Briefly, 1 g ALR was added to Tris–HCl solution to obtain 1% ALR staining buffer solution, followed by the addition of 1 g Tris–HCl to 100 ml distilled water. The pH of the solution was adjusted to 7.8 with 0.1 M HCl. Experimental and control groups of cells were incubated for 21 days. After washing twice with PBS buffer, the cells were then fixed with 95% ethanol for 10 min. After washing with PBS buffer again, the cells were incubated with 1% ALR staining buffer solution for 10 min at 37°C. In order to eliminate the non-specific bindings, the cells were incubated in 3 ml PBS solution for 30 min at room temperature and washed gently with PBS solution. The mineralization nodule formation was observed and photographed under an inverted fluorescence microscope. To semi-quantify the mineralization nodule formation, 10% cetylpyridinium chloride in 10 mM Na_2_HPO_4_ was added, followed by shaking for 10 min at room temperature. The absorbance was then measured at a wavelength of 562 nm using a microplate reader.

### 2.12. Statistical analysis

All data in graphs are generated from at least three independent experiments, and expressed as the means ± s.d. as indicated. Prism was used to evaluate the data for statistical significance by two-tailed Student's *t*-tests (figures 1,2,4*c*,5) and one-way ANOVA (figures 3,4*b*,6) with *p < 0.05 or ^#^*p* < 0.05 (versus the indicated controls) considered as significant.

**Figure 1.** TNF-α treatment upregulated miR-150-3p and downregulated β-catenin expressions in hBM-MSCs. (*a*) Expressions of miR-150-3p in hBM-MSCs treated with either PBS (as control) or TNF-α. (*b*) Expressions of several genes known to be regulated by TNF-α in hBM-MSCs after the same treatment as in (*a*). (*c*) Expressions of genes from (*b*) in hBM-MSCs transfected with either miR-NC (negative control) or miR-150-3p. Data were presented as mean ± s.d. from at least three independent experiments. **p < 0.01, *p < 0.05 compared with respective PBS or miR-NC control.

**Figure 2.** TNF-α treatment upregulated miR-150-3p, which directly targeted the 3′-UTR on β-catenin mRNA in hBM-MSCs. (*a*) Sequence of the putative miR-150-3p targeting site (capitalized nucleotides) on the 3′-UTR of β-catenin mRNA. (*b*) At the downstream of a luciferase reporter open reading frame (LUF), wild-type (-WT) or mutated (-Mut, grey nucleotides) versions of putative targeting sequence from the 3′-UTR of β-catenin mRNA were cloned. (*c*) Luciferase activities of LUF-WT and LUF-Mut constructs were measured in hBM-MSCs co-transfected with either miR-NC (negative control) or miR-150-3p. Data presented as mean ± s.d. from at least three independent experiments. **p < 0.01, *p < 0.05 compared with respective PBS or miR-NC control. (*d*) Luciferase activities of LUF-WT and LUF-Mut constructs were measured in hBM-MSCs treated with either PBS (as control) or TNF-α. (*e*) β-catenin protein levels in hBM-MSCs transfected with either miR-NC or miR-150-3p were examined by Western blot. (*f*) hBM-MSCs were transfected with either miR-NC or miR-150-3p inhibitor (anti-miR), and treated with either PBS (−) or TNF-α (+), followed by Western blot analysis to examined β-catenin protein levels.

**Figure 3.** IKK activation was essential for TNF-α induced upregulation of miR-150-3p in hBM-MSCs. (*a*) Expressions of miR-150-3p in hBM-MSCs treated with p38 MAPK inhibitor BIX02188, JNK inhibitor SP600125 and IKK inhibitor TPCA-1, respectively, in the presence of TNF-α. (*b*) NF-κB protein and (*c*) miR-150-3p levels in hBM-MSCs transfected with siRNAs against NF-κB were examined. (*d*) β-catenin protein levels in hBM-MSCs treated with small inhibitors (left panels) or siRNAs against NF-κB (right panels) in the presence of TNF-α were examined with Western blot. (*e*) Levels of phosphorylated NF-κB at Ser536 (p-NF-κB) in hBM-MSCs treated with either PBS (as control) or TNF-α. Data presented as mean ± s.d. from at least three independent experiments. **p < 0.01 compared with respective Mock or siRNA-NC control.

**Figure 4.** NF-κB-induced miR-150-3p expression by directly binding to its promoter region. (*a*) Promoter region of human miR-150 gene contains three putative binding sites for NF-κB. At the upstream of a luciferase reporter open reading frame (LUF), segments of putative NF-κB binding sites from the miR-150 promoter were cloned. (*b*) Binding of NF-κB to the promoter of miR-150 in hBM-MSCs was examined by ChIP assay using IgG (as control) or anti-NF-κB antibody. (*c*) Luciferase activities of ABC-LUF, BC-LUF and C-LUF constructs were measured in hBM-MSCs treated with either PBS (as control) or NF-κB. Data presented as mean ± s.d. from at least three independent experiments. **p < 0.01 compared with respective IgG or PBS control.

**Figure 5.** TNF-α treatment and miR-150-3p transfection both inhibited osteogenic differentiation of hBM-MSCs. (*a*) Calcium content, alizarin red (ALR) and alkaline phosphatase (ALP) staining assays were measured in hBM-MSCs treated with either PBS (as control) or TNF-α. (*b,c*) Representative images of ALR and ALP stainings (*b*), and expressions of Runx2 and Osx (*c*) after the same treatment as in (*a*). (*d*) Calcium content, alizarin red (ALR) and alkaline phosphatase (ALP) staining assays were measured in hBM-MSCs transfected with either miR-NC (negative control) or miR-150-3p. (*e,f*) Representative images of ALR and ALP stainings (*e*), and expressions of Runx2 and Osx (*f*) after the same treatment as in (*d*). Data presented as mean ± s.d. from at least three independent experiments. **p < 0.01, *p < 0.05 compared with respective PBS or miR-NC control.

**Figure 6.** MiR-150-3p was required for TNF-α-induced inhibition of hBM-MSC osteogenic differentiation. (*a*) hBM-MSCs were transfected with either miR-NC (as control) or miR-150-3p inhibitor (anti-miR), then treated with either PBS (as control) or TNF-α, followed by measurements of calcium content, alizarin red (ALR) and alkaline phosphatase (ALP) stainings. (*b,c*) Representative images of ALR and ALP stainings (*b*), and expressions of Runx2 and Osx (*c*) after the same treatment as in (*a*). For the easy of comparison, results from figure 5 (PBS and TNF-α treatments) were also plotted. Data presented as mean ± s.d. from at least three independent experiments. **p < 0.01, *p < 0.05 compared with respective PBS control. ##*p* < 0.01, #*p* < 0.05 compared with respective miR-NC control.

## 3. Results

### 3.1. TNF-α induces miR-150-3p expression and decreases β-catenin levels in hBM-MSCs

The mesenchymal stem cells derived from human bone marrow were isolated by a conventional protocol and used in the following study (electronic supplementary material, figure S1). We have confirmed the progenitor cell identity by the flow cytometry analysis of well-known surface markers in human mesenchymal stem cells, including positive markers CD29, CD105, CD90 and negative marker CD45 [23].

As a potential modulator of cell differentiation and bone matrix mineralization [24], we focused on miR-150-3p in hBM-MSCs during TNF-α treatment (table 2). As shown in figure 1*a*, 20 ng ml^−1^ TNF-α treatment on hBM-MSCs for 24 h induced a significant increase in miR-150-3p expression. As microRNAs function to suppress target genes, we next assessed the potential effects of miR-150-3p induction in hBM-MSCs. We examined the target genes that are known to be repressed by TNF-α (table 2), including peroxisome proliferator-activated receptor alpha (PPAR-α), intercellular adhesion molecule 2 (ICAM2), growth hormone receptor (GHR), CRH receptor-2 (CRH-R2), endothelial nitric oxide synthase (eNOS) and β-catenin [25–30]. Consistent with previous findings, we observed that TNF-α downregulated all these gene expressions in hBM-MSCs (figure 1*b*). Interestingly, in hBM-MSCs transfected with miR-150-3p, only β-catenin expression was decreased compared with the miR negative controls (figure 1*c*), suggesting that miR-150-3p induction by TNF-α might mediate the suppression of β-catenin in hBM-MSCs.

**Table 2.** Genes reported to be downregulated by TNF-α.

PPAR-α	peroxisome proliferator-activated receptor alpha [25]
ICAM2	intercellular adhesion molecule 2 [26]
GHR	growth hormone receptor [27]
CRH-R2	corticotropin releasing hormone receptor 2 [28]
eNOS	nitric oxide synthase [29]
β-catenin	catenin beta-1 [30]

### 3.2. TNF-α induced miR-150-3p targets the 3′-UTR of β-catenin mRNA

By computational analysis, we found a region of complementary sequence on the 3′-UTR of β-catenin predicted to bind miR-150-3p (figure 2*a*). Luciferase reporter assays were then performed to evaluate the specificity of the 3′-UTR of β-catenin for binding to miR-150-3p, by cloning wild-type or mutated versions of putative targeting sequence from the 3′-UTR of β-catenin mRNA to the downstream of a luciferase reporter open reading frame (figure 2*b*). As shown in figure 2*c*, co-transfection of miR-150-3p greatly decreased the luciferase activity of the construct with the wild-type 3′-UTR of β-catenin (WT), whereas the inhibition was completely abolished when the putative miR-150-3p binding sites were mutated (Mut). Similarly, TNF-α decreased the luciferase activity of WT 3′-UTR but not in the Mut-3′-UTR of β-catenin (figure 2*d*). Notably, the studies of the 3′-UTR reporter assays are relevant to *in vivo* gene regulation in hBM-MSCs, as β-catenin protein levels were clearly downregulated by either miR-150-3p (figure 2*e*) or TNF-α (figure 2*f*). We further pretreated cells with blocking oligonucleotides for miR-150-3p (anti-miR-150-3p). Consistently, compared with control oligos, the repression of β-catenin protein by TNF-α was prevented by anti-miR-150-3p (figure 2*f*). These data revealed an indispensable role of miR-150-3p for TNF-α inhibiting β-catenin, which was clearly mediated through binding of miR-150-3p to a complementary sequence on the 3′-UTR region of β-catenin mRNA.

### 3.3. NF-κB activation was required for miR-150-3p induction by TNF-α

We next explored the molecular mechanisms responsible for the increased miR-150-3p expression seen in hBM-MSC treated with TNF-α. The pharmacological inhibitors of several signalling pathways known to be activated by TNF-α were used, including p38 MAPK inhibitor BIX02188, JNK inhibitor SP600125 and IKK inhibitor TPCA-1, respectively. A significant blockade of miR-150-3p induction by TNF-α was only observed in cells treated with TPCA-1 (figure 3*a*). We then tested two sets of siRNAs targeting p65 NF-κB (figure 3*b*), and found that they both prevented the induction of miR-150-3p by TNF-α in hBM-MSCs (figure 3*c*), further supporting that IKK/NF-κB signalling might be essential for miR-150-3p upregulation by TNF-α. Furthermore, under the same IKK/NF-κB inhibitory conditions as figure 3*a*,*c*, we found that changes in primary miR-150 levels closely followed that of mature miR-150-3p (electronic supplementary material, figure S2), indicating the observed upregulation of mature miR-150-3p was indeed caused by enhanced transcription of pri-miR-150 by NF-κB. Indeed, in hBM-MSCs TNF-α increased p65 phosphorylation (figure 3*e*), a marker for IKK/NF-κB signalling activation. Using the repression of β-catenin protein by TNF-α as an alternative readout of miR-150-3p induction, we found that blocking either IKK by TPCA-1 or NF-κB by siRNAs could prevent the decrease of β-catenin protein (figure 3*d*).

A direct binding of NF-κB to the promoter region of miR-150 was then investigated. The upstream promoter region of human *miR-150* gene (miRBase Accession MI0000479) was retrieved from GeneBank annotation (NC_000019.10: 49,499,285-49,500,785). We found that there are three potential NF-κB-responsive DNA-binding sites bearing the consensus sequences-GGRNNYYC (where R is purine, Y is pyrimidine T C and N is any base), and named them A (−1057), B (-686) and C (−94) regions, respectively (figure 4*a*). In ChIP assays performed in hBM-MSCs, a specific binding of NF-κB to B region in the promoter of miR-150 was highlighted, as compared with other regions or control IgG immunoprecipitations (figure 4*b*). Consistent with the specific requirement of the binding sites for miR-150 induction, the transcriptional activity of the miR-150 promoter stimulated by NF-κB was lost when B region was truncated (figure 4*c*). Taken together, our above results clearly indicate that NF-κB activation was essential for the miR-150-3p induction following TNF-α treatment in hBM-MSCs.

### 3.4. TNF-α inhibited osteogenic differentiation of hBM-MSCs through miR-150-3p

Maintenance of β-catenin protein is important for driving osteoblast differentiation, maturation and mineralization. To elucidate whether downregulation of β-catenin by TNF-α can alter osteogenesis in hBM-MSCs, we examined the differentiation markers of osteoblast, namely calcium contents, alizarin red (ALR) and alkaline phosphatase (AP) activities, and specific gene expressions (figure 5). As expected, TNF-α treatment on hBM-MSCs inhibited the ALR and ALP activities, decreased calcium contents (figure 5*a*,*b*) and reduced the gene expressions of bone formation markers (Runx2 and Osterix in figure 5*c*).

Similarly, hBM-MSCs transfected with miR-150-3p showed an attenuated osteogenic differentiation, manifested by decreased ALR, ALP, calcium contents and Runx2/Osterix expressions (figure 5*d–f*), consistent with our previous findings that miR-150-3p also decreased β-catenin (figures 1 and 2). To determine whether miR-150-3p was indispensable for the suppressive effects of TNF-α on osteogenic differentiation, anti-miR-150-3p was used to treat cells in the presence of TNF-α treatment. Compared with control oligos, hBM-MSCs transfected with anti-miR-150-3p were resistant to TNF-α treatment (figure 6). Transfection of scrambled control miR in hBM-MSCs did not affect the inhibition of osteogenesis by TNF-α, whereas miR-150-3p transfection protected the reductions in calcium contents, ALR and ALP activities (figure 6*a,b*). Additionally, the declines of Runx2 and Osterix expressions in TNF-α-treated cells were reversed only in the presence of antisense oligonucleotides to miR-150-3p (figure 6*c*). Our data strongly demonstrated that TNF-α inhibition on osteogenic differentiation of hBM-MSCs was mediated through upregulation of miR-150-3p expression.

## 4. Discussion

In this study, we discovered miR-150-3p as a novel regulator in mediating osteogenesis inhibition by TNF-α. Through a newly identified NF-κB-binding site on the promoter of miR-150, TNF-α directly stimulated miR-150-3p expression. The importance of miR-150-3p has then been demonstrated by both gain-of-function and loss-of-function studies. The overexpression of miR-150-3p mimicked, whereas anti-miR-150-3p prevented, TNF-α-induced inhibition of osteogenic differentiation in hBM-MSCs. Finally, the function of miR-150-3p may depend on modulating β-catenin levels in hBM-MSCs. miR-150-3p targeted on the 3′-UTR of β-catenin to decrease its expression. These data collectively featured miR-150-3p as a potentially important post-transcriptional regulator of osteogenesis in the context of inflammation.

MicroRNAs have emerged as an important class of gene modulators. However, their functions have yet to be unravelled. The best characterized functions of miR-150-3p thus far mainly included the regulations on haematopoietic cell development. For instance, by targeting a transcription factor c-Myb controlling lymphocyte development, miR-150-3p modulates the differentiation of B cells, natural killer (NK) cells and invariant NK T (iNKT) cells [31,32]. In addition, miR-150-3p expression was upregulated in inflammatory conditions such as sepsis with a wide spectrum of putative gene targets in immune cells [33]. Consistently, our studies identified a direct NF-κB binding site at the miR-150 promoter region, and data in hBM-MSCs have suggested that TNF-α/IKK/NF-κB signalling, the major pro-inflammation pathway, can directly activate miR-150-3p expression (figures 1 and 4). This is particularly interesting, as increased proinflammatory signalling cascades suppress bone formation activity, as evident in facture healing, osteoporosis and rheumatoid arthritis [2,3,5]. Our novel findings that miR-150-3p is a direct target of TNF-α, combined with the previous observations that miR-150-3p can block cell terminal differentiation, implied that miR-150-3p may act as a major microRNA involved in immunosuppression of bone cell regeneration. In support of this hypothesis, we found that transfection of miR-150-3p reduced the osteogenic differentiation in hBM-MSCs (figure 5). However, the roles of miR-150-3p in osteoblast differentiation are still unclear and have been confounded by conflicting data in recent investigations. Studies in an *in vitro* bone formation model using mouse osteoblastic cell line MC3T3-E1 have suggested that miR-150-3p expression promoted bone matrix mineralization [24]. By contrast, overexpression of miR-150-3p did not affect osteoblast differentiation of pre-osteoblast cells derived from neonatal mouse calvaria [34]. It is not known if loss of miR-150-3p could affect bone formation. MiR-150-3p knockout mice exhibited decreased bone mass, but mainly due to increased osteoclast activities [34]. Together these differences may suggest diverse functions of miR-150-3p in modulating bone formation processes, depending upon the various stages of osteoblast development influenced by distinct cellular contexts. Our data clearly showed that miR-150-3p expression could antagonize *in vitro* osteogenesis of hBM-MSCs. The physiological relevance of this finding may be further tested by investigating embryonic bone development or postnatal bone repair models in miR-150-3p knockout animals.

The molecular basis of TNF-α induced miR-150-3p expression is consistent with a conventional transactivation of miRNA genes that depends on NF-κB p65. A classic NF-κB signalling stimulated by inflammatory cytokines such as TNF-α includes the activation of IκBα kinase (IKK) pathway, the nuclear translocation of p65, and induced transcription activation of its target genes. A variety of microRNAs contain the canonical NF-κB responsive element in the promoter regions [35–37]. In our studies, a direct binding of NF-κB p65 subunit to the promoter of miR-150 (-686 from the start site) was demonstrated by ChIP assays (figure 4*b*). The regulation of miR-150 promoter by NF-κB was subsequently confirmed by a reporter assay with truncated binding sites (figure 4*c*). Inhibition of NF-κB with an IKK inhibitor blocked miR-150-3p stimulation by TNF-α (figure 3). Interestingly, alterations in miR-150-3p expression were readily observed during inflammatory responses as a potential immune suppressor [33,38]. For instance, miR-150-3p was found to target MyD88 [39], a critical adaptor protein found in many TNF-α receptor-associated signalling complexes, suggesting that miR-150-3p may act as a negative feedback regulator of TNF-α signalling.

β-catenin is essential for Wnt signalling in promoting osteogenic differentiation and cancer development [12]. It has been shown that microRNAs could modulate Wnt/β-catenin in different scenarios of tumour progression. MiR-200a was found to directly inhibit β-catenin mRNA translation in meningioma cells [40]. Overexpression of miR-122 decreased the protein levels of β-catenin in hepatocellular carcinoma [41]. On the other hand, microRNAs may activate β-catenin. MiR-374a expression in metastatic breast cancer cells constitutively activated β-catenin signalling by the downregulation of Wnt/β-catenin suppressor such as PTEN [42]. MiR-26a-mediated GSK-3β destruction has been found to be able to induce β-catenin levels in cholangiocarcinoma [43]. To identify related microRNAs, a systemic approach was employed to dissect the involved microRNAs in Wnt signalling pathway during *in vitro* cell differentiation such as adipogenesis [44]. Here we identified another novel microRNA that negatively regulated β-catenin signalling. More specifically, miR-150-3p induction by TNF-α in hBM-MSCs was found to inhibit β-catenin-dependent osteogenic differentiation. As previously discussed, miR-150-3p could be one of the important endogenous determinators of osteogenesis, similarly as other candidate microRNAs that play regulatory roles in Wnt/β-catenin pathway in osteoblastic differentiation [19,20]. More significantly, our data suggested that miR-150-3p was at a nexus of osteogenesis, β-catenin signalling and inflammation stimuli TNF-α. There are multiple levels of co-regulations between β-catenin and TNF-α signalling. The same E3-ubiquitin ligase, the SCF complex, mediates the destructions of IκBα and β-catenin with opposite effects on downstream signalling. The targeted degradation of IκBα activates the subsequent NF-κB nuclear functions, while the destabilization of β-catenin prevents its roles in transcription co-activation. β-catenin could physically bind with NF-κB, leading to decreases of NF-κB DNA-binding and target gene expression [30]. It was also shown that TNF-α enhanced β-catenin stabilization during early adipogenesis [45]. The present data have identified an additional player in this setting, namely miR-150-3p, which mediated negative impact of TNF-α signalling on β-catenin. Such regulation may be responsible for the diminished osteoblast activity that occurs in a series of inflammatory bone diseases. Our findings may also provide mechanistic insights for the link between inflammation and pathogenesis of cancer, in which both β-catenin and miR-150-3p have been intimately associated with the origin, progression and metastasis of tumours. Investigation of this issue in miR-150-3p knockout mice will be of particular interest to study if the potential increase of β-catenin activity would contribute to tumourigenesis.

## 5. Conclusion

In summary, we have investigated the potential functions of microRNAs for modulating osteogenesis during inflammation. In human bone marrow mesenchymal stem cells, miR-150-3p, a major modulator of immunity, negatively affected osteogenic differentiation through decreasing β-catenin. By directly stimulating miR-150-3p expression through NF-κB activation, TNF-α inhibited β-catenin-dependent osteogenesis of mesenchymal stem cells. Thus, our work uncovered a novel mechanism for TNF-α-induced inhibition of bone formation activity, which could be used as a therapeutic target for the treatment of inflammatory bone diseases.

## Supplementary Material

Supplementary Materials
